The article "Deep Learning-Based CT Imaging to Evaluate the Therapeutic Effects of Acupuncture and Moxibustion Therapy on Knee Osteoarthritis" was published in 2022. Journal: Comput Math Methods Med.

# Deep Learning-Based CT Imaging to Evaluate the Therapeutic Effects of Acupuncture and Moxibustion Therapy on Knee Osteoarthritis

**DOI:** 10.1155/2022/1135196

**Published:** 2022-05-21

**Authors:** Guoyong Jiang, Jianguang Ding, Chenglu Ge

**Affiliations:** ^1^Department of Chinese Medicine, Changyi People's Hospital, Changyi, 261300 Shandong, China; ^2^Department of Critical Medicine, Changyi People's Hospital, Changyi, 261300 Shandong, China; ^3^Department of CT, Changyi People's Hospital, Changyi, 261300 Shandong, China

## Abstract

The study was aimed at analyzing the application value of deep learning-based computed tomography (CT) in evaluating the effect of acupuncture for knee osteoarthritis (KOA). Specifically, 124 patients with KOA were selected in the test group (warm acupuncture and moxibustion) and the control group (simple acupuncture), with 62 cases in each group. Deep learning-based CT scanning was performed before and after treatment to compare the Lequesne-Mery, Visual Analog Scale (VAS), Western Ontario and McMaster Universities (WOMAC), Hospital Special Surgery (HSS), and Knee Society Score (KSS) scores as well as the overall effective rate. The results showed that the trabecular thickness, quantity, bone mineral density (BMD), connection density, structural model index, and articular cartilage thickness were different significantly between the two groups (*P* < 0.05). After treatment, the Lequesne-Mery was 4.78, the VAS was 0.87, and the WOMAC score was 14.89 of the test group, which were reduced (*P* < 0.05). The KSS and HSS scores of the test group were improved significantly after treatment (*P* < 0.05). The total effective rate of the test group was 85.48%, and that of the control group was 51.61%; the former was significantly higher than the latter (*P* < 0.05). In conclusion, acupuncture could improve the clinical effect on KOA patients, and CT scanning under deep learning algorithm could evaluate the clinical effect of acupuncture for KOA.

## 1. Introduction

Knee osteoarthritis (KOA) is a disease characterized by progressive articular cartilage degeneration and plate reactive bone loss [1]. Inflammation, local injury, and chronic knee strain can all lead to KOA; patients often experience joint pain and even disability, which has a serious impact on the quality of life [2–5]. Researches have shown that KOA is strongly associated with obesity, gender, and genetics. Middle-aged and older adults are primarily affected by KOA. Secondary KOA is usually caused by a variety of joint diseases, including joint injuries, fractures, joint fractures, and joint ligament strains [6–8]. According to statistics, 3% of people in China suffer from KOA. When the age is over 55, the incidence of KOA can reach 60%; and when the age is over 65, the incidence of KOA increases again, reaching over 80% [9–11]. The occurrence and development of KOA pathological processes are complex and unclear. Studies have shown that it starts from the degenerative changes of knee articular cartilage, gradually affects the subchondral plate and joint capsule, and finally leads to the progressive destruction of articular cartilage and synovial inflammation [12]. Patients with KOA always have clinical symptoms such as joint pain, swelling, and mobility impairment [13–15]. KOA is classified as joint pain in traditional Chinese medicine. *The Yellow Emperor's Internal Canon of Medicine* believes that the combination of wind, cold, and dampness can lead to bone diseases. Knee pain is due to liver and kidney impairment caused by cold and dampness [16]. The symptoms of joint pain described in the classic literature are consistent with KOA symptoms, including knee swelling [17, 18]. The application of acupuncture has a long clinical history in the treatment of bone diseases [19]. Acupuncture can help relieve pain, relax tendons, activate meridians, and eliminate aseptic inflammation and local edema of knee joint, as well as dredge meridians in patients [20–22].

Computed tomography (CT) is a commonly used method for clinical evaluation of the severity of KOA patients. Compared with X-ray, CT has advantages for its high sensitivity and avoiding the effects of overlap or artifacts during X-ray. In addition, CT can present the specific conditions of bone lesions in a more detailed and perfect manner [23–25]. Clinical workers often cannot summarize from CT image quantitative, accurate medical information by the naked eye, while the medical image analysis and processing technology solves this dilemma. By reading extremely complex impact information from CT images and establishing corresponding algorithms for further analyses, clinicians can more accurately and quickly diagnose the disease and obtain more in-depth information about the disease [26, 27]. Convolutional neural network is a deep neural network with a deeper structure. It can convert image data into visual pathological features and discover feature data that cannot be obtained by naked human eyes [28].

In this study, the application value of deep learning-based CT was explored and analyzed in evaluating the effect of acupuncture for KOA. 124 patients with KOA were selected as the research objects, including 62 cases in the test group (warm acupuncture and moxibustion) and the other 62 cases in the control group (simple acupuncture). Deep learning-based CT scanning was performed before and after the treatment, to obtain imaging quantitative parameters. The scores of Lequesne-Mery, Visual Analog Scale (VAS), Western Ontario and McMaster Universities (WOMAC), Hospital Special Surgery (HSS), and American Knee Society Score (KSS) were compared between the two groups. As the total effective rate was also compared, the effect of acupuncture for KOA was evaluated. By studying the evaluation effect of deep learning-based CT on the effect of acupuncture in the treatment of KOA, it was expected to provide treatment options for KOA patients.

## 2. Materials and Methods

### 2.1. Research Objects

In this study, 124 patients with KOA who were treated from February 2, 2018, to June 2, 2021, were selected as the research objects. These patients were divided into a test group and a control group, with 62 cases in each group. Those in the test group were treated with warm acupuncture and moxibustion, while those in the control group were treated with simple acupuncture only. The patients included in this study signed the informed consent forms, and the research process had been approved by the ethics committee of hospital.

Inclusion criteria: (I) patients diagnosed with KOA per diagnostic criteria of traditional Chinese and Western medicine, (II) the patient was in good condition without other serious organ diseases, (III) patients who cooperated in CT examination, (IV) patients without any test contraindications, and (V) patients who had not accepted related treatment related to this study.

Exclusion criteria: (I) patients with knee joint tumor, (II) patients with gouty arthritis, (III) patients with mental diseases unable to cooperate in acupuncture treatment and efficacy evaluation, (IV) pregnant or lactating patients, and (V) patients whose family members did not agree or did not sign the informed consent.

### 2.2. CT Examination

CT was performed on all patients using 16-slice spiral CT scanner. The patients were scanned in the supine position, and the scanning range was from the proximal tibia to the distal femur, including the entire knee joint; and an axial scanning was taken. Specific scanning parameters included the tube voltage 120 kV, the tube current 70 mA, the layer thickness 5 mm, and the layer spacing 5 mm. Scannings were performed at 0.37 seconds at 360°, and 20 images were reconstructed per second.

### 2.3. Deep Learning Algorithm

ResNet, as an excellent object detection, image classification, and segmentation model, has been widely used in convolutional neural networks. Residual structures in the ResNet model make it easier to optimize. In the propagation process of neural network, the propagation gradient often disappears gradually due to the occurrence of back propagation. However, the residual structure solves this problem, and the gradient information of residual structure is more easily transmitted in the process of back propagation. Its specific structural model is shown in Figure 1.

The original convolutional kernel of inception structure is decomposed from 5×5 and 7 × 7 into 5 × 1 and 1 × 5 and 7 × 1 and 1 × 7. To avoid the disappearance of gradient information during back propagation, ResNet residual structure is combined with inception model. Feature information in inception network images is extracted and the result *t* is output to complete the global average pooling. To reduce the number of *t* channels and reduce calculation parameters, the results obtained in the previous step will pass through the full connection layer, so as to update the result to *T*_1_ × *t*. Through the assignment of nonlinear layer activation function, the activation function result is output, which is expressed as *F*. The result is continuously input to the fully connected layer, and another parameter *E* is introduced to output the result *E*_2_*F*(*T*_1_ × *t*), so as to reduce channel number. Next, the results obtained in the previous step are further delivered to the nonlinear layer, and then, the weight data of the above channels are obtained. Finally, all information parameters are collected in the full connection layer. The corresponding information of two models (ResNet and inception) is superimposed, and the ResNet residual model is only combined with inception in the last step, as shown below.

(1) $$\begin{array}{c} N=R\left(E_{2}F\left(T_{1}\times t\right)\right). \end{array}$$

### 2.4. Acupuncture and Moxibustion Therapy

In the test group, patients were treated with warm acupuncture and moxibustion. The patients were in a supine position, with the knee joints naturally bent. The acupuncture sites (Dubi, Liangqiu, Xuehai, and Zusanli acupoints) were disinfected. Then, 2 cm needle was inserted into the meridians. After qi was invigorated by neutral supplementation and draining, the needle was retained in the appropriate depth. Three acupoints were selected in total. Subsequently, 2 cm moxa stick was lit. Warm acupuncture and moxibustion was given once every two days, with 6 times as a course, a total of two courses. In the treatment process, the patient should stay in a warm environment, have a balanced diet, and avoid fatigue.

The control group received simple acupuncture treatment: the needle was inserted directly at the acupoint site with a depth of about 3 cm. After qi was invigorated by neutral supplementation and draining, the needle was retained for 30 min and then removed, and alcohol cotton ball was pressed for disinfection.

### 2.5. Observation and Evaluation Indicators

General basic data, including mean age, male to female ratio, course of disease, and size of tibial plateau, were collected and compared between the two groups.

The Lequesne-Mery score of knee joint is as follows: rest pain, tenderness, movement pain, swelling pain, and morning stiffness score 0-3 and walking ability scores 0-6, with a total score of 23. The total effective rate of the two groups after treatment was evaluated: 0-2 is considered as cured, 3-8 as remarkably effective, 9-18 as effective, and 19-23 as ineffective. The total effective rate *M* is calculated according to Equation (2), wherein the total number of patients is *S*, the cured number is *R*, and the remarkably effective number is *X*.

(2) $$\begin{array}{c} M=\frac{S+R}{X}\times 100\%. \end{array}$$

VAS, WOMAC, HSS, and KSS are measured before and after treatment in the two groups.

### 2.6. Statistical Methods

SPSS17.0 was applied for statistical analysis of data. Normally distributed data were presented as mean ± standard deviation ($\bar{x}\pm s$), *t*-test was adopted to represent measurement data, and chi-square (*χ*^2^) test was used to represent enumeration data. *P* < 0.05 represents statistical difference.

## 3. Results

### 3.1. Basic Information of Patients

The basic data of patients were not different significantly between the two groups, in terms of average age, gender distribution, and course of disease (*P* > 0.05), which are shown in Figure 2. This indicated the comparability between the two groups.

The sizes of tibial plateau and tibial angle were recorded and compared between the two groups, and the results showed no significant difference between the two groups (*P* < 0.05), indicating comparability between the two groups, as shown in Figure 3.

### 3.2. CT Imaging Data

Figure 4 displays CT images of male patients with different KOA. The results showed that the patients started to develop osteophytes, the joint space narrowed gradually compared to that of normal people, and sclerotic changes appeared. Joint hypertrophy and obvious deformity could be observed.

### 3.3. Imaging Parameters

CT imaging scan based on deep learning algorithm was performed to obtain the relevant parameters of patients in the two groups before and after treatment. The results showed that there were significant differences in trabecular thickness, trabecular number, and bone mineral density (BMD) between the two groups after treatment (*P* < 0.05), but no significant differences in trabecular septum (*P* > 0.05), as shown in Figure 5.

In addition, compared with those of the control group, the connection density and structural model indicators were remarkably increased in the test group after treatment (*P* < 0.05), which are shown in Figure 6.

Before treatment, articular cartilage thickness comparison results showed no significant difference between the two groups of patients (*P* > 0.05). As shown in Figure 7, the articular cartilage thickness in the test group was highly increased after treatment compared with that in the control group (*P* < 0.05). Besides, the thickness after treatment was greater than that before treatment in the test group (*P* < 0.05).

### 3.4. Lequesne-Mery, VAS, and WOMAC Scores and the Effective Rate

Lequesne-Mery, VAS, and WOMAC scores were measured before and after treatment, and the effective rate was calculated. As presented in Figures 8 and 9, all these scores were greatly decreased after treatment in the test group compared with those in the control group (*P* < 0.05). The total effective rates were also significantly different between the two groups after treatment (*P* < 0.05).

### 3.5. KSS and HSS Scores

The KSS and HSS scores of patients in the two groups were recorded, mainly in pain, motion, muscle strength, stability, and other aspects. The scores of HSS and KSS in the test group were higher significantly than those in the control group (*P* < 0.05), which could be found in Figure 10.

## 4. Discussion

With the rapid development and progress of science and technology and medical technology, the population aging is becoming increasingly serious, and the incidence of KOA is increasing year by year. KOA is caused by the joint action of mechanical and biological factors, manifests as the broken balance of subchondral bone, chondrocytes, and extracellular matrix, and leads to progressive articular cartilage degeneration and bone growth at joint edges [29, 30]. KOA is common in middle-aged and elderly people. With the aging of the population and the increase of obesity rate, the prevalence of KOA keeps climbing to a new height. At present, there are more than 100 million KOA patients in China [31]. Clinically, the disease is usually manifested as knee joint swelling, pain, limited joint activity, stiffness, reduced stability, and even joint configuration and dysfunction in severe cases, which greatly affects patients' quality of life [32]. Traditional Chinese medicine says when healthy qi is weak and the liver, spleen, and kidney are deficient, exogenous pathogenic factors of wind, coldness, and dampness invade the body to block qi and blood. Thus, the treatment should be based on the principle of tonifying liver and kidney, promoting blood circulation, dredging meridians, and relieving pain. The application of acupuncture and moxibustion therapy in the treatment of bone diseases has a long clinical history. Acupuncture and moxibustion therapy can help patients with analgesia, relax tendons and activate meridians, eliminate aseptic inflammation and local edema of the knee joint, and realize the purpose of dredging the meridians [33]. In this study, warm acupuncture and moxibustion therapy was used to treat KOA and its therapeutic efficacy was evaluated.

In this work, the application value of deep learning-based CT was analyzed in evaluating the effect of acupuncture for KOA. The imaging quantitative parameters, obtained by CT scanning under deep learning before and after treatment, were compared between the test group (warm acupuncture and moxibustion) and the control group (simple acupuncture). The Lequesne-Mery, VAS, WOMAC, HSS, and KSS scores were compared as well as the total effective rate between the two groups. There was no significant difference between the two groups in average age, gender distribution, course of disease, size of tibial plateau, and tibial angle (*P* > 0.05). CT scanning parameters suggested the significant differences in trabecular thickness, trabecular number, and BMD between the two groups after treatment (*P* < 0.05), but no significant difference was shown in trabecular spacing (*P* > 0.05). Compared with the control group, the connection density and structural model index of the test group increased notably after treatment (*P* < 0.05). The articular cartilage thickness of the test group also increased (*P* < 0.05), and that after treatment was significantly higher than that before treatment (*P* < 0.05). These indicated that all CT scanning parameters greatly changed after treatment in both groups, and CT scanning deserved the application value in evaluating the effect of acupuncture and moxibustion. Furthermore, the Lequesne-Mery, VAS, and WOMAC scores of the test group were significantly decreased after treatment in comparison with those in the control group (*P* < 0.05), and the total effective rate of the test group was highly increased (*P* < 0.05). The KSS and HSS scores of the test group were better than those of the control group, indicating that acupuncture could improve the clinical symptoms of KOA patients, promote deep learning-based CT scanning, and evaluate the clinical effect on KOA. The introduction of CT scanning results into the evaluation system of the severity and treatment effect on KOA patients showed a good application effect. As CT scannings were performed on KOA patients before and after treatment, it was proved that CT scanning parameters could determine the treatment effect comprehensively, which was consistent with the findings of this work [34, 35]. In short, deep learning-based CT images were of great significance for the effect evaluation of KOA patients after acupuncture treatment. Acupuncture could improve the clinical effect on KOA patients and also was worthy of popularization and application.

## 5. Conclusion

In this work, the application value of deep learning-based CT was analyzed for the effect evaluation of acupuncture in the treatment of KOA. It was demonstrated that acupuncture therapy could improve the clinical symptoms of KOA patients, and deep learning-based CT scanning could evaluate the clinical effect on KOA better. However, the disadvantage of this work lay in the small sample size, so the findings are needed to be further verified. During follow-up, it was necessary to expand the sample size to strengthen the results.

## Figures and Tables

**Figure 1:** Structure of ResNet model.

**Figure 2:** Comparison of the basic conditions of the two groups of patients. (a), (b), and (c) showed the gender distribution, average age, and course of disease, respectively.

**Figure 3:** Tibial plateau and tibial angle in the two groups.

**Figure 4:** CT images of KOA patients. (a) was of the patient 1, male, 37 years old; (b) was of the patient 2, male, 45 years old; (c) was of the patient 3, male, 42 years old; and (d) was of the patient 4, male, 43 years old.

**Figure 5:** Comparison of related parameters between the two groups after treatment. (a) The trabecular thickness and spacing. (b) The BMD and trabecular number. ^∗^Compared to the control group, *P* < 0.05.

**Figure 6:** Comparison of structural model index and connection density parameters between the two groups after treatment. (a) Structural model index. (b) Connection density. ^∗^Compared to the control group, *P* < 0.05.

**Figure 7:** Comparison of articular cartilage thickness between the two groups before and after treatment. ^∗^Compared to the control group, *P* < 0.05.

**Figure 8:** Comparison of scores between the two groups before and after treatment. (a) VAS. (b) WOMAC. (c) Lequesne-Mery. ^∗^Compared to the control group, *P* < 0.05.

**Figure 9:** Comparison of effective rates between the two groups after treatment. ^∗^Compared to the control group, *P* < 0.05.

**Figure 10:** Comparison of HSS and KSS scores between the two groups. (a) HSS score. (b and c) KSS score. ^∗^Compared to the control group, *P* < 0.05.

## Data Availability

The data used to support the findings of this study are available from the corresponding author upon request.

## References

[1] Bennell K. L., Paterson K. L., Metcalf B. R. (2021). Effect of intra-articular platelet-rich plasma vs placebo injection on pain and medial tibial cartilage volume in patients with knee osteoarthritis: the RESTORE randomized clinical trial. *Journal of the American Medical Association*.

[2] Patel V. G., Oh W. K., Galsky M. D. (2020). Treatment of muscle-invasive and advanced bladder cancer in 2020. *CA: a cancer journal for clinicians*.

[3] Onwunzo C. N., Igwe S. E., Umunnah J. O., Uchenwoke C. I., Ezugwu U. A. (2021). Effects of isometric strengthening exercises on pain and disability among patients with knee osteoarthritis. *Cureus*.

[4] Chung H. K., Wen S. H., Chang W. C., Liu K. L. (2021). Acute surgical site infection after total knee arthroplasty in patients with rheumatoid arthritis versus osteoarthritis. *Scientific Reports*.

[5] Jin T., Cheng Z. X. (2021). Current status and thoughts of non-surgical treatment of knee osteoarthritis. *Zhonghua Yi Xue Za Zhi*.

[6] Bucci J., Chen X., LaValley M. (2022). Progression of knee osteoarthritis with use of intraarticular glucocorticoids versus hyaluronic acid. *Arthritis & Rheumatology*.

[7] Sharma S., Wilson R., Pryymachenko Y. (2021). Reliability, validity, responsiveness, and minimum important change of the stair climb test in adults with hip and knee osteoarthritis. *Arthritis care & research*.

[8] Marouf B. H. (2021). Effect of resveratrol on serum levels of type II collagen and aggrecan in patients with knee osteoarthritis: a pilot clinical study. *BioMed Research International*.

[9] Bi X., Li T., Li M. (2021). A new method to develop the primate model of knee osteoarthritis with focal cartilage defect. *Frontiers in Bioengineering and Biotechnology*.

[10] Shamsi M., Safari A., Soroush A., Safari Y. (2021). The survey of knee osteoarthritis in the population over age 50 visited in the health bus in Kermanshah, Iran. *Journal of aging research*.

[11] Yeoh P. S. Q., Lai K. W., Goh S. L. (2021). Emergence of deep learning in knee osteoarthritis diagnosis. *Computational Intelligence and Neuroscience*.

[12] Fu S., Duan T., Hou M. (2021). Postural balance in individuals with knee osteoarthritis during stand-to-sit task. *Frontiers in Human Neuroscience*.

[13] Wu R., Ma Y., Yang Y., Li M., Zheng Q., Fu G. (2022). A clinical model for predicting knee replacement in early-stage knee osteoarthritis: data from osteoarthritis initiative. *Clinical Rheumatology*.

[14] Aoyagi K., Liew J. W., Farrar J. T. (2022). Does weight-bearing versus non-weight-bearing pain reflect different pain mechanisms in knee osteoarthritis?: the multicenter osteoarthritis study (MOST). *Osteoarthritis and Cartilage*.

[15] Li S. M., Li T. L., Guo R. (2021). Effectiveness and safety of acupotomy for knee osteoarthritis: study protocol for a randomized controlled trial. *Trials*.

[16] Sun Q., Zhang K., Chen J., Xu Y., Liu Y., Zheng R. (2020). Traditional Chinese medicine classification of knee osteoarthritis with proteomics analysis. *Annals of Palliative Medicine*.

[17] Li R., Chen H., Feng J. (2020). Effectiveness of traditional Chinese exercise for symptoms of knee osteoarthritis: a systematic review and meta-analysis of randomized controlled trials. *International Journal of Environmental Research and Public Health*.

[18] Zhou X., Xiang K., Yuan X., Wang Z., Li K. (2020). Chinese herbal medicine Wutou decoction for knee osteoarthritis: a protocol for systematic review and meta-analysis. *Medicine (Baltimore)*.

[19] Xu X., Wan Y., Gong L., Ma Z., Xu T. (2020). Chinese herbal medicine Yanghe decoction for knee osteoarthritis: a protocol for systematic review and meta-analysis. *Medicine*.

[20] Wu Y. Y., Bai M., Tian S., Miao M. S. (2020). Animal model analysis of knee osteoarthritis based on clinical characteristics of Chinese and Western medicine. *Zhongguo Zhong Yao Za Zhi*.

[21] Lo P. C., Lin F. C., Tsai Y. C., Lin S. K. (2019). Traditional Chinese medicine therapy reduces the risk of total knee replacement in patients with knee osteoarthritis. *Medicine*.

[22] Gu Y. G., Jiang H. (2019). Correlation between synovitis and traditional Chinese medicine syndromes of knee osteoarthritis in WORMS score. *Zhongguo Gu Shang*.

[23] Roemer F. W. (2021). Weight-bearing CT for knee osteoarthritis assessment: a story unfolds. *Radiology*.

[24] De Laroche R., Simon E., Suignard N. (2018). Clinical interest of quantitative bone SPECT-CT in the preoperative assessment of knee osteoarthritis. *Medicine (Baltimore)*.

[25] Flynn C., Hurtig M., Lamoure E. (2020). Modeling and staging of osteoarthritis progression using serial CT imaging and arthroscopy. *Cartilage*.

[26] Kim J., Lee H. H., Kang Y. (2017). Maximum standardised uptake value of quantitative bone SPECT/CT in patients with medial compartment osteoarthritis of the knee. *Clinical Radiology*.

[27] Sumida Y., Nakasa T., Ishikawa M., Nakamae A., Adachi N. (2021). The evaluation of degeneration of posterior cruciate ligament using CT Hounsfield unit in knee osteoarthritis. *BMC Musculoskeletal Disorders*.

[28] Tsukada A., Uchida K., Aikawa J. (2020). Unilateral-dominant reduction in muscle volume in female knee osteoarthritis patients: computed tomography-based analysis of bilateral sides. *Journal of Orthopaedic Surgery and Research*.

[29] Nissen N., Holm P. M., Bricca A., Dideriksen M., Tang L. H., Skou S. T. (2022). Clinicians' beliefs and attitudes to physical activity and exercise therapy as treatment for knee and/or hip osteoarthritis: a scoping review. *Osteoarthritis and Cartilage*.

[30] Joseph G. B., McCulloch C. E., Nevitt M. C., Link T. M., Sohn J. H. (2022). Machine learning to predict incident radiographic knee osteoarthritis over 8 years using combined MR imaging features, demographics, and clinical factors: data from the osteoarthritis initiative. *Osteoarthritis and Cartilage*.

[31] Yeh H. W., Chan C. H., Yang S. F. (2022). Total knee replacement in osteoarthritis patients on reducing the risk of major adverse cardiac events: a 18-year retrospective cohort study. *Osteoarthritis and Cartilage*.

[32] Iuamoto L. R., Imamura M., Sameshima K., Meyer A., Battistella L. R., Fregni F. (2021). Functional changes in cortical activity of patients submitted to knee osteoarthritis treatment: an exploratory pilot study. *American Journal of Physical Medicine & Rehabilitation*.

[33] Yang M., Jiang L., Wang Q., Chen H., Xu G. (2017). Traditional Chinese medicine for knee osteoarthritis: an overview of systematic review. *PLoS One*.

[34] Perlman A., Fogerite S. G., Glass O. (2019). Efficacy and safety of massage for osteoarthritis of the knee: a randomized clinical trial. *Journal of general internal medicine*.

[35] Rajendran K., Murthy N. S., Frick M. A. (2020). Quantitative knee arthrography in a large animal model of osteoarthritis using photon-counting detector CT. *Investigative Radiology*.

